# Retrospective Study of the Application Value Analysis of Ultrasound-Guided Technology in Peripheral Deep Venous Catheterization of Neonates

**DOI:** 10.1155/2022/1726906

**Published:** 2022-07-23

**Authors:** Tingting Yin, Yuan Huo, Yang Zhao, Weiyang Li, Hongxia Gao

**Affiliations:** Neonatal Department, Gansu Provincial Maternity and Child-Care Hospital, 143 Qilihe North Street, Lanzhou City, Gansu Province, China 730050

## Abstract

**Objective:**

To investigate the application value analysis of ultrasound-guided technology in peripheral deep venous catheterization of neonates.

**Method:**

A total of 94 neonates who underwent peripheral deep venous catheterization treatment from March 2020 to August 2021 in our hospital were selected and divided into the study group and the control group according to the simple randomized method, and each group had 47 cases. The control group was performed peripheral deep venous catheterization through X-ray examination, while the study group was performed peripheral deep venous catheterization through ultrasound-guided technology. The catheter placement, catheter retention time and adjustment times, the incidence of complications (limb swelling, pain, fluid leakage, and phlebitis), and the intervention satisfaction of family members were counted.

**Results:**

The success rate of one-time catheterization in the study group was higher than that in the control group, the operation time was shorter than that in the control group, and the amount of bleeding was less than that in the control group. The indwelling time of catheter in the study group was longer than that in the control group, and the number of adjustments was less than that in the control group. The incidence of complications in the study group was lower than that in the control group. The intervention satisfaction of family members in the study group was higher than that in the control group.

**Conclusion:**

Peripheral deep venous catheterization in neonates through ultrasound-guided technology can reduce operation time and blood loss and ensure the success rate of one-time catheterization, resulting in a long indwelling time of catheter, low number of adjustments, and low incidence of complications, which has safety and high intervention satisfaction of family members.

## 1. Introduction

Peripherally deep vein catheterization is a technique to establish venous access by positioning the tip of the catheter in the vena cava through the peripherally deep vein. It can safely infuse irritant drugs, which is of great significance to reduce pain and protect blood vessels. It is convenient for medical staff to implement relevant treatment and nursing operations and has been widely used in clinic [1, 2]. Peripheral deep venous catheterization plays an important role in neonatal pediatrics. It can provide a good foundation for the treatment of preterm infants and ultralow/very low birth weight infants and create a venous pathway for the successful treatment of children [3].

The end position of peripheral deep venous catheterization is of great significance to ensure the effectiveness and safety of treatment. If the insertion length is too short or too deep, it may cause chemical phlebitis, and arrhythmia and other serious adverse events may occur in severe cases [4]. Therefore, how to ensure the safety and efficacy of peripheral deep venous catheterization is still the hotspot.

In the past, peripheral deep vein catheterization was assisted by X-ray examination, which was simple and easy, but X-ray examination had certain radiation damage, and the organs of newborns were not yet mature, so it was easy to cause varying degrees of damage to neonates [5]. In recent years, the application value of ultrasound-guided technology in the diagnosis and treatment of a variety of diseases has been widely recognized. The implementation of peripheral deep vein catheterization under ultrasound guidance can ensure the success rate of catheterization and avoid radiation injury [6]. However, there are few systematic studies on the application value of ultrasound-guided peripheral deep vein catheterization in neonates. Based on this, 94 neonates who received peripheral deep vein catheterization in our hospital were selected to explore the application value of ultrasound-guided technology.

## 2. Material and Methods

### 2.1. General Information

A total of 94 neonates who underwent peripheral deep venous catheterization treatment from March 2020 to August 2021 in our hospital were selected and divided into the study group and the control group according to the simple randomized method, and each group had 47 cases. There were 26 males and 21 females in the study group. Gestational age ranged from 26 to 41 weeks, with an average of 33.34 ± 4.61 weeks. The average age was 14.64 ± 6.22 days. The birth weight was 1261.5~4694.7 g, with an average of 2978.06 ± 307.66 g. The puncture sites were the external jugular vein in 1 case, head vein in 2 cases, lower limb vein in 4 cases, and upper limb vein in 40 cases. There were 28 males and 19 females in the control group. The gestational age ranged from 25 to 41 weeks, with an average of 33.08 ± 5.05 weeks. The average age was 15.10 ± 5.97 days. The birth weight was 1237.6~4711.2 g, with an average of 3006.54 ± 298.96 g. The puncture sites were the external jugular vein in 1 case, head vein in 1 case, lower limb vein in 6 cases, and upper limb vein in 39 cases. The clinical data of the two groups such as gender, day age, gestational age, birth weight, and puncture site were balanced and comparable (*P* > 0.05), and this study was approved by the ethics committee of our hospital.

### 2.2. Selection Criteria

The inclusion criteria were as follows: (1) the family members of the patients were aware of the study and signed a paper consent form, (2) there is an indication of peripheral deep venous catheterization, and (3) no other central venous access was inserted before catheterization. The exclusion criteria were as follows: (1) bleeding tendency and hemorrhagic disease, (2) coagulation dysfunction, (3) infection or trauma in the route of intubation, (4) death before normal extubation, (5) and patient's family member voluntarily withdrawal during the study period.

### 2.3. Treatment

For the patients in the control group, the peripheral deep vein catheterization was assisted by X-ray examination. The equipment was a MOBILETT XP digital X-ray camera of Siemens company in Germany to carry out photographic positioning. The catheter was placed to the predicted length, and then, the guide sheath was withdrawn for hemostasis and fixation. For the patients in the study group, the catheter was placed through the peripheral deep vein with the help of ultrasound-guided technology. The equipment selected the LOGIQ E color Doppler ultrasound diagnostic instrument of GE company of the United States. The catheter tip was positioned through the ultrasound-guided technology, the catheter was placed to the predicted length, the guide sheath was not removed temporarily, and the ultrasound examination was carried out. The ultrasound image showed that there was a bright shadow at the inlet of the right atrium of the inferior or superior vena cava; then, 1 ml of normal saline was injected. The vortex different from the normal blood flow can be seen through the ultrasonic image. After clarifying the catheter tip was about 10~20 mm at the opening of the right atrium of the inferior or superior vena cava, the guide sheath was withdrawn for hemostasis and fixation.

### 2.4. Observation Indexes

(1) The catheterization situation between the two groups was counted, including the one-time catheterization success rate, operation time, and blood loss. (2) The catheter indwelling time and adjustment times of the two groups were counted. (3) The incidence of complications in the two groups includes swelling, pain, fluid leakage, and phlebitis. (4) The intervention satisfaction of family members between the two groups was counted. The self-made satisfaction scale was used to evaluate the catheterization and skin condition at the puncture site by the patient's family members. A total of 100 points were obtained. 90~100 points were very satisfied, 70~89 points were basically satisfied, and less than 70 points were dissatisfied. Total satisfaction = (remarkable effect + effective)/total number of cases × 100%.

### 2.5. Statistical Analysis

SPSS22.0 was used for statistical analysis; measurement data was expressed as $\bar{x}\pm s$ and analyzed by a *t*-test. The enumeration data was expressed as *n* (%) and analyzed by *χ*^2^ test. *P* < 0.05 indicated that the difference was statistically significant.

## 3. Results

### 3.1. Comparison of Catheter Placement between the Two Groups

As shown in Table 1, the success rate of one-time catheterization in the study group (97.87%) was higher than that in the control group (85.11%), the operation time 3.04 ± 0.95 min was shorter than that in the control group 8.69 ± 1.94 min, and the amount of bleeding 1.11 ± 0.34 ml was less than that in the control group 1.79 ± 0.40 ml; the differences were statistically significant (*P* < 0.05).

### 3.2. Comparison of Indwelling Time of Catheter and the Number of Adjustments between the Two Groups

The indwelling time of the catheter in the study group was (17.39 ± 2.58 days) longer than that in the control group (10.37 ± 1.49 days), and the number of adjustments (1.53 ± 0.30 times) was less than that in the control group (2.35 ± 0.39 times); the differences were statistically significant (*P* < 0.05, Table 2).

### 3.3. Comparison of the Incidence of Complications between the Two Groups

The incidence of complications in the study group (4.26%) was significantly lower than that in the control group (19.15%) (*P* < 0.05, Table 3).

### 3.4. Comparison of the Intervention Satisfaction of Family Members between the Two Groups

The intervention satisfaction of family members in the study group (95.74%) was significantly higher than that in the control group (82.98%) (*P* < 0.05, Table 4).

## 4. Discussion

Peripheral deep venous catheterization is widely used in neonatal central venous pressure monitoring, central venous administration, parenteral nutrition support, and so on. It plays an important role in the treatment of neonates in the intensive care unit [7]. However, the peripheral blood vessels of newborns are usually thin, some of which are variable, or are difficult to reach, which can easily lead to puncture failure [8]. Therefore, how to improve the success rate of peripheral deep vein catheterization is still a research hotspot.

The traditional puncture method of peripheral deep vein catheterization is mainly to puncture and withdraw according to the anatomical marks on the body surface and evaluate whether the puncture is successful according to the color and pressure of the extracted blood. If the pressure is small, there is no obvious fluctuation, and the blood is dark red, it may be a vein; if the pressure is large, the fluctuation is obvious, and the blood is bright red, it may be an artery. After a successful puncture, the guide wire is inserted, the skin expander is used to expand the skin, and the venous catheter is inserted along the guide wire. However, the puncture success rate of this mode is low, it is easy to puncture the artery by mistake, and multiple punctures are very easy to damage the tissue, so the clinical application has limitations [9, 10]. It has been reported that the incidence of mechanical injury in patients with traditional central venous catheterization can reach 5%~19%, which is mainly related to nerve injury, air embolism, arteriovenous fistula, hemopneumothorax, hematoma formation, wrong puncture of artery, and other complications [11, 12]. Although the peripheral deep vein puncture and catheterization assisted by X-ray film can improve the success rate to a certain extent, it is difficult to show the radiation injury of blood vessels during the examination, and the catheter displacement cannot be corrected. The catheter displacement can only be determined according to bone identification and venous anatomical positioning. The neonatal blood vessels are not fully developed, and it is difficult to accurately determine the location [13, 14]. Ultrasound is also an important clinical examination technology. Some studies have pointed out that through ultrasound examination technology, dynamic development can be realized to accurately identify the vascular structure. Through ultrasonic positioning, the status of the catheter in the vein can be dynamically and clearly displayed. During catheter placement, the limb abduction angle can be adjusted in real time, and the position of the catheter tip can be dynamically monitored to ensure that it reaches the preset position, so as to ensure the accuracy of positioning and puncture and prevent complications such as catheter displacement to the greatest extent [15, 16].

Our study has suggested that the success rate of one-time catheterization in the study group was higher than that in the control group; the operation time, the amount of bleeding, and the number of adjustments in the study group were lower than those in the control group; the indwelling time of catheter in the study group was longer than that in the control group; the incidence of complications in the study group was lower than those in the control group; and the intervention satisfaction of family members in the study group was higher than that in the control group, indicating that ultrasound-guided technology in peripheral deep venous catheterization of neonates has a high application value and can reduce operation time and ensure accuracy and safety of puncture catheterization, thus reducing the incidence of complications. The reason is that peripheral deep venous catheterization through ultrasound-guided technology can develop, monitor, and adjust the catheter displacement in real time and prevent the catheter tip from being placed too deep or too shallow, and there is no need to reconstruct the sterile area or catheter secondary fixation, which is conducive to optimizing the operation process, reducing the stimulation of repeated adjustment of the catheter tip position on neonatal blood vessels, and reducing the occurrence of related complications [17, 18]. At the same time, the neonates need to be moved with the help of X-ray examination, and the temperature fluctuation and radiation damage caused by leaving the incubator are easy to cause adverse effects on neonates. Ultrasonic examination has the advantages of simple operation and no need to move the newborn repeatedly, and there is no interruption of treatment and nursing [19]. In addition, neonatal limb adduction and abduction will affect the catheter position, and changes in arm posture, elbow extension, and flexion will also affect the catheter position. Such changes are difficult to be detected by X-ray film, and ultrasound can provide real-time information and avoid ray injury [20, 21]. This study has found that the success rate of peripheral deep venous catheterization through ultrasound-guided technology was still less than 100%, which may be due to the younger age of neonates, crying caused by treatment stimulation, examination and pain caused by disease, decreased coordination, and improper body position during puncture, which would affect the results of ultrasound-guided localization, thus leading to puncture failure.

In summary, peripheral deep venous catheterization in neonates through ultrasound-guided technology can reduce operation time and blood loss and ensure the success rate of one-time catheterization, resulting in a long indwelling time of catheter, low number of adjustments, and low incidence of complications, which has safety and high intervention satisfaction of family members. However, this study is a single-center small sample study, which is also its limitation. It possibly led to a certain bias in the conclusions of this study. Therefore, it is still necessary to further confirm the above conclusions by clinical multicenter and large sample studies.

## Figures and Tables

**Table 1:** Comparison of catheter placement between the two groups.

Groups	Cases	Success rate (*n*, %)	Operation time (min)	Bleeding (ml)
Study	47	46 (97.87)	3.04 ± 0.95	1.11 ± 0.34
Control	47	40 (85.11)	8.69 ± 1.94	1.79 ± 0.40
*χ* ^2^/*t* value		3.937	17.932	8.880
*P* value		0.047	0.001	0.001

**Table 2:** Comparison of indwelling time of catheter and the number of adjustments between the two groups.

Groups	Cases	Indwelling time of catheter (d)	Number of adjustments (times)
Study	47	17.39 ± 2.58	1.53 ± 0.30
Control	47	10.37 ± 1.49	2.35 ± 0.39
*t* value		16.153	11.425
*P* value		0.001	0.001

**Table 3:** Comparison of the incidence of complications between the two groups.

Groups	Cases	Limb swelling	Pain	Fluid leakage	Phlebitis	Incidence
Study	47	0 (0.00)	1 (2.13)	1 (2.13)	0 (0.00)	2 (4.26)
Control	47	1 (2.13)	4 (8.51)	2 (4.26)	2 (4.26)	9 (19.15)
*χ* ^2^ value						5.045
*P* value						0.025

**Table 4:** Comparison of the intervention satisfaction of family members between the two groups.

Groups	Cases	Very satisfied	Basically satisfied	Dissatisfied	Total satisfaction
Study	47	29 (61.70)	16 (34.04)	2 (4.26)	45 (95.74)
Control	47	25 (53.19)	14 (29.79)	8 (17.02)	39 (82.98)
*χ* ^2^ value					4.029
*P* value					0.045

## Data Availability

The authors confirm that the data supporting the findings of this study are available within the article.
